# Impact of Social Media on Geopolitics and Economic Growth: Mitigating the Risks by Developing Artificial Intelligence and Cognitive Computing Tools

**DOI:** 10.1155/2022/7988894

**Published:** 2022-05-11

**Authors:** M. M. Kamruzzaman

**Affiliations:** Department of Computer Science, College of Computer and Information Sciences, Jouf University, Sakakah, Saudi Arabia

## Abstract

Social media is one of the most revolutionary innovations in computer science that facilitates connecting people in the world to share information, ideas, and thoughts. In recent years, social media has demonstrated tremendous growth, which has affected individuals, businesses, communities, and economies. The focus of the present study is to identify the impact of social media on geopolitics and economic growth. The study is based on a systematic review of previous literature on the subject. It has been revealed through the findings that social media impacts geopolitics by decreasing the level of censorship and increasing the spread of news or information, while it also enables the politicians to influence individuals over online social networks through the great level of access. On the other hand, it has been identified that social media has both positive and negative impacts on geopolitics and economic growth. Social media is able to unite diverse groups and individuals spread across the planet dedicated to specific issues. The formation of communities and the ability of social media to unite groups show how social media could contribute positively to geopolitics and economic growth. But it decreases the productivity level of the individuals; on the other hand, it does contain the potential to create a participatory economy, which can be beneficial for a particular country. Some argue that social sharing has encouraged people to use computers and mobile phones to express their concerns on social issues without actually having to engage actively with campaigns in real life. Their support is limited to pressing the “Like” button or sharing content. This study performs a thorough study selection exercise and a quality assessment to ensure that the present study is valuable to academia and the relevant stakeholders, especially the experts of computer science who can develop the smartest artificial intelligence and cognitive computing tools that can help mitigate those risks of social media for the geopolitically volatile, uncertain, complex, and ambiguous world and ensure smooth economic growth.

## 1. Introduction

The advent of multidisciplinary research was inspired by the growing demand of social relations and computer-mediated communication since the mid 1980s. Social media has seen a massive rise in the late 2000s. More specifically, the previous decade has observed a significant evolution in its forms and usage [1]. The range of features that this technology offers attracts a wide range of consumers. According to [2], social media can be defined as being computer-mediated technologies developed by the expert of computer science that are interactive in nature and are able to facilitate the sharing or creation of information, career interests, and ideas in addition to other forms of expression through networks and communities that are virtual.

The present study aims to analyze the impact of social media on geopolitics and economic growth and how to mitigate the risks by developing artificial intelligence (AI) and cognitive computing tools. The topic is relevant as social media's growth has a pivotal impact on the political and business environments at the micro and macro levels [2]. Due to its complexity and vast usage, there is no formula or specific technique on how to run social media accounts successfully. Thus, companies and other governmental agencies have adopted a personalized tactic for handling social media to obtain favourable results. According to [3], social media is used by businesses in the United Kingdom for the purpose of product promotion, driving sales, recruitment, brand awareness, forming networks, and customer service. This states that there is a vast range of operations for social media platforms. From a political perspective, the concept of “geopolitics” is relevant here. Geopolitics is equivalent to normal politics, yet defined by international boundaries and international relations influenced by geographical factors [4].

AI is the simulation of human intelligence, processed and exhibited by machines. The underlying idea is to enable computer systems to perform tasks in line with human intelligence, via a set of theories, methods, and algorithms, whereas cognitive computing is a subfield of AI and refers to computing that focuses on reasoning and understanding at a higher level. Computing is analogous to human cognition, rationale, and judgment. It has the capacity to deal with symbolic and conceptual information. It is receptive to different kinds of stimuli and is able to take accurate decisions in complex situations. AI and cognitive computing are key components of the popular social networks, which we use every single day. Facebook uses advanced machine learning (ML) to do everything to recognize photos to target users with advertising. Instagram uses AI to identify visuals. LinkedIn uses AI to offer job recommendations, suggest people you might like to connect with, and serve you specific posts in your feed. Snapchat leverages the power of computer vision, an AI technology, to track your features and overlay filters that move with your face in real time. And, across all social media platforms and each social media post, an AI algorithm or machine learning system is regulating how the content you create and the ads you buy are placed in front of users—often in ways that are not entirely transparent to marketers.

There are multiple types of social media platforms; the most prominent ones used are microblogging, product review system websites, social networking sites, and blogs [5]. Microblogging websites, such as Twitter, are meant for users to share their thoughts in a limited number of words. These websites are used by companies, government agencies, local shops, and so on for marketing, announcing, or just providing information for the users. A direct link is created between the two factions, which is a good opportunity for both parties to communicate their needs and issues [5]. Product review system websites are meant for consumers and companies to access to check the feedback of other users of certain products, whereas social networking sites are the key social media platforms, which are the most popular among users. The most prominent example of this type of social media platform is Facebook. Due to the vast number of users, companies and other agencies find it convenient to communicate via social media about new offerings. The last type is blogs, which are used by individuals mostly for multiple purposes, yet most prominently for giving out opinions about multiple topics such as fashion, politics, and so on [2].

Moreover, there are multiple uses of social media; however, it is used in specific ways by organizations. Some of these uses are communication, marketing, promotion, and research [6]. Communication has been made very easy by social media platforms, and thus, it is no surprise that users apply social media for effective communication. Direct connection is established between two parties, which is not possible with traditional forms of mass communication platforms such as TV advertising [6]. Marketing, which is a process of value creation for a product or service, is significantly pursued via social media nowadays. Here, branding is a well-known example, where businesses establish social media profiles and share relevant content to promote their brand. Market research, which is a component of a product/service's marketing, is a key factor that social media is used. Social media has made it convenient for researchers to conduct market research as more trends can be identified, including the identification of consumer preferences and purchase intention [7].

The present study is essential for multiple reasons; firstly, politics and social media have a mixed relationship as the two entities often do not match the motives [8]. For example, the motive of politics to influence their opinions and slogans among the vast population may not be deemed ethical by the social media platforms as they may be responsible for propaganda or wrongful agendas. Furthermore, the issue of fake news is a huge area of concern from the political aspect as it may harm the campaign of politicians in the wrong way [9]. For example, fake news spread on social media regarding a price hike on a commodity may cause an outrage, which was not even caused by the governing entities. Therefore, politics and social media are a very delicate mix. The present study's findings can enable academia and experts of different domains to have clearer answers towards the relationship between the geopolitics and social media for developing new theory and smart artificial intelligence (AI) and cognitive computing tools that will be used in social media similar to AI and cognitive computing tools that have been extensively used to leverage individual behaviours, preferences, beliefs, and interests to personalize experiences and to find where you have been, where you are going, what you have written in emails, what you have asked your voice assistants, what groups you belong to, what stores you shop at, and more.

Like businesses, politicians are now also bound to social media as it allows them to communicate with the subjects as they intend [10]. A lot of famous political personalities have made social media accounts to gain an advantage through good publicity [11]. Due to its complex nature, political organizations construct proper strategies to use social media to their advantage. However, things do not always work out according to the plans; for example, Facebook refused ads from multiple American presidential candidates in the 2016 election as the ads did not meet their community standards [12]. Therefore, it is required for political entities to be fairly responsible on social media since they are bound to influence a large number of people.

Previous research suggests that geopolitics contains the essential elements of international relations, which can be influenced by social media as the activities of a country's political entity are public [13]. Inappropriate use of social media, such as careless exchange of content might hurt public sentiments or affect deals. It is observed that political personalities of different nations often exchange words on social media platforms, especially Twitter [14]. Wrongful or aggressive contact among different nations' individuals can cause a spur of reaction among individuals, often leading to local news channels covering the spat and causing a negative environment. A recent example of the exchanges on Twitter between political heads of America and Iran has caused a wide range of spur leading to protests and outrage [15]. Therefore, it is understood that the link between geopolitics and social media could have very adverse consequences and should be dealt with utmost care.

Economic growth can be represented by many factors; most prominently, it is represented by the GDP growth or GDP per capita growth [16]. It is observed that economic growth is influenced by four main factors, which include human capital, physical capital, and availability and quantity of natural resources and technology. Human capital corresponds to the labour and the population of a country. An efficient workforce of the country can add value to economic growth; however, an unskilled or poorly developed workforce can cause damage to the growth and could potentially give rise to unemployment [17]. Physical capital refers to the infrastructure of the country as it helps develop the materials and other commodities for growth. The availability and quantity of natural resources available in a country can determine the level of dependency it will have on other nations. On the other hand, technology is a referral point for economic growth for a lot of countries as more advanced technologies enable the country to apply a better method for production and economic growth [16].

The present research is essential in regard to the topic of economic growth as social media falls under the technology category as an influencer of economic growth. Reference [18] states that, in general, there is a negative link between social media and economic growth. However, when control variables are introduced (such as marketing), social media can influence economic growth positively [19]. Economic growth can be influenced by social media, where factors such as promotion and fake news can intrigue buying behaviour, among other elements. A country's fake news can lead to a lesser investment or tourism, leading to a hit to economic growth [19]. Therefore, the present study can enable practitioners and policymakers to achieve a deeper understanding of social media's impact on economic growth and develop AI and cognitive computing tools that can help mitigate the risks of social media and keep smooth economic growth. It performs a systematic review to achieve the objectives and provides an overview or synthesis of the available evidence.

Geopolitics and economic growth elements can be interlinked in a lot of ways. Political setting can influence economic growth in a positive or negative way [20]. Healthy relations between the two countries can increase the level of trade, leading to higher economic growth [21]. Furthermore, certain indicators/factors such as interest rate, exchange rate, tariffs, and taxes can also be used to form a relationship between the two variables [22]. Moreover, geopolitics and economic growth can be affected by indicators such as ease of doing index. If the political determination of these factors is favourable, then it would be more likely that economic growth would be high due to added investment from other countries.

On the other hand, if geopolitical conditions are not favourable, then there would likely be discrepancies in the economy of the country [20]. The example of Afghanistan could be relevant here, which struggles from the poor geopolitical situation due to unfriendly relations with the neighbouring countries and poor local management [23]. Here, social media may play its role in influencing both the geopolitical outlook and economic growth of the country. In the following section of the study, the methodology applied to execute the study is presented.

As indicated earlier, the methodology used in this study is a qualitative systematic review, while AMSTAR and PRISMA tools are applied. AMSTAR is applied to identify the quality of the research by undertaking the questions generated by the tool, whereas the PRISMA tool is applied to narrow down the studies used in the research for review.

The rest of the study is systematically organized such that first the methods used are comprehensively discussed by defining key elements such as the research approach and design, literature search, study selection, quality assessment, and data extraction and analysis. Furthermore, the results are portrayed, and the discussion is presented based on those results. Finally, the conclusion is given based on the overall findings of the present study.

## 2. Materials and Methods

### 2.1. Research Approach and Design

The present study applies a qualitative approach; however, it assumes a positivist philosophy since it aims to identify the impact of social media on geopolitics and risks to economic growth. The study has been selected to be qualitative as it satisfies the aim of the research. The researcher seeks in-depth knowledge of the issue while not depending on numerical data for statistics. Furthermore, keeping the descriptive nature of qualitative studies in mind would help interpret a wide range of literature that include journal articles. For this purpose, the study adopts a systematic review approach. The review method was established prior to the conduct of the review. Moreover, there is no external funding involved in this study.

### 2.2. Literature Search

The systematic qualitative approach is taken by the review of journal articles and other secondary sources with a similar topic. The articles correspond to the topic, that is, the impact of social media on geopolitics and risk on economic growth. It means that the literature search involved various related keywords, including social media and geopolitics, social media and economic growth, impact of social media on geopolitics and economic growth, and artificial intelligence. The articles searched are from 2011 to 2019 so that the studies applied are not outdated. They are extracted from numerous sources, including Google Scholar, Springer, Elsevier, Emerald, and EBSCOhost, to ensure that the studies are credible and authentic.

### 2.3. Study Selection

This paper analyzes a total of 10 most relevant studies. The journal articles that reported the impact of social media on geopolitics and economic growth are included based on the following criteria:

- The articles must be published during the selected period, that is, from 2011 to 2021
- The articles must have sufficiently addressed the research problem, that is, the article is relevant to the study
- The articles include information regarding the influence of social media on either economic growth or geopolitics or both
- Articles selected must be from credible journals
- The articles must have a clearly written abstract with conclusions and methodological implications
- The structure of the studies must be defined clearly, along with transparency in the research approach, a predefined technique and process, discussion of literature, sample size, and documented clearly conclusions
- References are included in the present study to ensure that the credit for the study goes to the authors, while the present study remains credible

### 2.4. Quality Assessment

AMSTAR tool is used in the present study for performing a quality assessment of the paper. AMSTAR has been categorized as a reliable and valid tool by [24] for assessing a systematic review's methodological quality. AMSTAR was applied in the present study by undertaking a survey provided by the tool, and in turn, the tool gave its assessment of the quality. Quality assessment is shown in Table 1, which has been rated as “moderate” by the online assessment tool.

### 2.5. Data Extraction and Analysis

PRISMA approach was taken to ensure that the present study remains of high quality and credible [25]. PRISMA approach is applied as this method ensured that relevant material was selected for the present study. PRISMA tool helps the researcher remove inappropriate or irrelevant research in order to form a good collection of studies to conduct the review.

The journal articles that satisfy the predefined requirements of selection are then also analyzed based on certain factors such as the publishing year, methods and tools applied for finding and testing, and geographical location of publishing. A narrative research design is then applied to analyze the findings of the study, while a systematic qualitative review is done for the selected studies for drawing the evaluations.

The following chart (Figure 1) illustrates the PRISMA procedure as it is applied in the present study:

With the help of the PRISMA procedure, the studies are selected that are the most relevant to the topic, have addressed the research problem, are wholly accessible, and meet the quality criteria identified in Section 2.3. Therefore, 15 main journals are reviewed in the present study. The main reason for the less number of studies short-listed for the systematic review was the issue of relevance since the research was unable to find the positive and/or negative impacts of social media on geopolitics and economic growth in the majority of the studies initially selected for review.

## 3. Results

The rise of social media should intrigue businesses into adopting social media in their global political risk management strategies as stated by [26]. The study states that “just in time” or targeted political risk management is not as effective as a multihazard approach where political risks are evaluated for a broader margin related to social media. Furthermore, the study states that a good political risk management plan can enable the business to cope with a volatile business environment. Moreover, the study states that social media influences geopolitics through an increased amount of protests. Lastly, the study proposes that good political risk management involves three elements. Firstly, chain resiliency procedures and plans shall be provided by a business in case of current business interruption. Secondly, an entity should be able to communicate potential problems to customers, employees, and suppliers. Thirdly, an organization should review its credit control procedures and policies and credit risks and make necessary adjustments [26].

Reference [27] states that due to the interconnectedness of the social media platforms, an opportunity is created for the participatory economy. A participatory economy can induce economic growth as more people get involved in contributing to the growth due to new opportunities created by social media. The participation of individuals on social media benefits quite a few other individuals; this creates new and unexpected results [27]. Moreover, the impact of social media on economic growth depends on the type of information and perception that is prevalent about certain products or companies in the market, which will determine their future growth [27].

The emergence of businesses from social media can be beneficial on the economic grounds, while it also has an impact on social relations and the well-being of individuals in a particular area. Conversely, in the study of [18], it is identified that social media has a significant and negative impact on economic growth. The article states that one of the reasons why the relationship between the two elements is negative is because the productivity of the individuals can be affected poorly by social media. The study rejected its hypothesis, which suggested that social media had a positive impact on economic growth [18]. The study possessed some drawbacks, such as the measurement errors relating to the existing proxies of social media technology and users' states. Further research suggestions included accessing whether the negative impact is due to greater consumption of nonmonetary content, decreased productivity, increased search costs, or a mix of the three factors.

Internet penetration and social media have positive impacts on economic growth. It contributes 3.2% of GDP in India and 4% of GDP in European countries. The reason behind this positive contribution is the social network is consumer-focused as well as a cost-effective marketing tool. So social media enables businesses to improve their product quality as well as product development planning [28]. It is also observed that social media don't have any significant impact on the economic development of the poorest communities but have a positive impact on developed economies [29]. Moreover, [28] also observed a positive link between social media and economic activities.

According to [30], social media has made some key changes that affect the political environment. Firstly, the users can comment or influence others regarding a political issue by being anonymous. Furthermore, there is a diversity and richness of information available on social media that can be used for or against political entities. Another change is the speed of how fast the news spreads; this can be negative for geopolitics as governments like to cease some information for their own benefit [30]. Another change is moving the society on social media from objectivity to subjectivity; issues are addressed for a longer period of time on social media as compared to digital media due to its vast space and presence [30]. Another change that can influence geopolitics is the ability of social media to influence users based on the combination of videos/images and text, which can be edited by any individual. Furthermore, censorship cannot prevent the whole issue as it can be done in other forms of traditional media; some parts of the news or other censored item can be accessed by individuals through social media. In reference [30], the ability of politicians to influence users and do effective campaigning has been stressed. Furthermore, it has been identified that political opponents at the national and international levels can use social media to learn from each other much more easily and openly.

A study by Aouragh and Chakravartty [31] states that through the formation of new communities and factions formed through social media, the political influence is carried and is embraced by individuals' part of communities. Furthermore, a rise in protests due to social media has also been linked in reference [31] for the political sense. Furthermore, the study stresses that sensitive political issues are discussed more openly on social media as compared to other digital media platforms, which impact geopolitics as governments like to censor some sort of information in order to preserve their image. However, the research of Chausovsky [32] states that the use of social media is influenced by geopolitics rather than the other way around. The study states that social media has the potential to act in political development, while it has already done so. However, the study states that impact is limited and cannot be a subject to carry out revolutions, while, ushering in regime change following these revolutions, social media simply serves as one tool among many as a force for political change [32]. Furthermore, it is discussed in the study that geopolitics can influence the usage of social media, as the regions such as Russia and China restrict the usage of foreign social media networks while making their own products for their people. Nonetheless, some form of exposure and escape from restrictions is found by social media users, even in strict Internet usage regions. The article further emphasizes the fact that social media has influenced political decisions, yet it does not possess the power for causing something as big and significant as a revolution [32].

In the study by Simons [33], it is stated that social media and new media are playing a greater part in international relations and politics. They are being used as a means to defend the existing world order and as a means to undermine it. These new forms of media are potentially very potent instruments of influencing the course and discussions on the existing world order and its possible directions. They are able to unite diverse groups and individuals spread across the planet dedicated to specific issues [33]. It has been stated that social media is being used by politicians to spread their message and not engage individuals. However, the messages received by the individuals are to be self-interpreted and acted upon accordingly [33].

Engesser et al. [34], in their study, link populism and social media and portray how politicians use social media as populists. The study states that politicians have the power to influence individuals on social media by adopting certain strategies that compliment populism [34]. Social media has provided a strong opportunity to populist politicians as they can reach a high number of people by using attractive content. Five key elements of populism were derived by [34] from the literature: advocating for the people, emphasizing the sovereignty of the people, ostracizing others, attacking the elite, and invoking the “heartland.” The qualitative studies revealed that populism presented itself in a fragmented form on social media. The study also states that populist politicians are given much more freedom on social media to express themselves and spread their ideas. The research conducted by [34] has given an opportunity in the future for better measurement and refined conceptualization of populism, especially regarding populism in social media.

It has been found in the study by Crilley and Gillespie [35] that a lack of accountability from social media outlets can cause the political use of social media to be out of control. The political use of social media platforms is conducted on unethical grounds and should be subject to appropriate restrictions. Reference [35] states that journalism has been harder due to social media that is influenced by populist politicians. The study states that due to few restrictions and open accessibility, the politicians can influence individuals on the social media platforms easily, which may be unethical on some grounds. Furthermore, the study states that a huge amount of data available on social media platforms of users can be used in politics by individuals to their advantage. The research further states that social media has made earnings for journalism harder, causing negative economic growth in that particular sector. The study suggests that there should be more restrictions on the use of social media by politicians to their advantage as it creates security concerns for the users [35].

In the study by Kiuru and Inkinen [36], it is found that there is a relationship between economic growth and social media; however, the relationship is negative as it has been observed that cities with fewer social media activities have a better growth from an economic point of view. Productivity is a measure that has been applied to multiple types of research to identify economic growth [36]. A decrease in productivity due to social media represents a decrease in the economic growth of a certain area. However, the study states that innovation leads to better economic growth, while the growth of social media can potentially be damaging to economic growth [36].

The geopolitical impact is further emphasized by [37] and [38], where it is observed that data-driven social media has both pros and cons in modern societies. Nations tightly control their information to express deterrence in modern geopolitics, which reflects the existence of negative consequences. Although it can be argued that social media do not have any revolutionary effects that change political systems, it does have evolutionary effects. Social media has helped raise movements against corruption and authoritarianism.

A summary of the findings made from the 10 studies in the present research is given in Table 2.

## 4. Discussion

### 4.1. Positive Impacts of Social Media on Geopolitics

Kay and Freely [26] state the rise of social media in recent years should intrigue the businesses adopting social media into their global political risk management strategies. This statement is supported in reference [39], who further states that businesses applying social media in their political risk management can create social value for the organization, which is a positive effect.

Moreover, the paper by [33] discusses in a political sense that social media platforms are being used as a means to defend the existing world order and as a means to undermine it. The use of social media has also been discussed in a similar tone in the study of [40]. While [33] also discusses that social media platforms are able to unite diverse groups and individuals spread across the planet dedicated to specific issues [41]. The formation of communities and the ability of social media to unite groups regarding issues are also stated in [26, 31]. It shows how social media could contribute positively to geopolitics. In addition, social media has positive effects on transforming the dynamics of geopolitics. It has changed the centre of power from the state to the individuals. Moreover, social media has mobilized society and created awareness in society that challenges oppressive regimes and brings a significant shift in geopolitics. The dynamics of the new world order are getting increasingly dependent on social media [33].

### 4.2. Negative Impacts of Social Media on Geopolitics

In the context of negative implications, it is observed that the political effect is carried and is incorporated by individuals' part of communities through the formation of new communities and factions formed through social media, as stated in the study of [31]. This statement is supported in the study of [10]. Furthermore, the study stresses that sensitive political issues are discussed more openly on social media as compared to digital media that impacts geopolitics as governments like to censor some sort of information in order to preserve their image. The limited censorship topic has been discussed in other studies [30]. Furthermore, a rise in protests is caused regarding politics through social media, as discussed in [15, 26], which may highlight the negative role of social media in terms of promotion of political instability and violence.

Furthermore, reference [34] states that on social media, politicians have the power to influence individuals by adopting certain strategies that compliment populism. Populism use of politicians in social media to influence followers has also been discussed in [35]. While the research of [34] further states that to express themselves and spread their ideas, populist politicians are given much more freedom on social media. This has been deemed as being negative in the study of [30] as the intentions of some politicians may not be in line with those of the individuals being influenced.

However, [26] reveals that social media influences geopolitics through an increased amount of protests; this claim has been supported in multiple studies such as [15, 31]. Furthermore, the study presents three key points that state what organizations can do to have better political risk management; these points can be used by multiple entities for achieving a good political risk management program based on long-term thinking.

The research by [30] reveals that due to social media, there have been multiple changes in the social environment, which can be used in the political sense. The most prominent change that occurred due to social media can be the ability of politicians to use social media to influence individuals towards an agenda, which favours their interests; this claim is also made in reference [8]. Furthermore, the article states that there is a range of information on social media, and the news spreads very fast over the platforms, as stated in reference [42]. Reference [30] also states that geopolitics is affected as the ability to censor content on social media is limited as compared to other forms of media. Reference [43] also states a similar observation regarding information spread and geopolitics.

It is observed that a lack of accountability from social media outlets can make the political use of social media out of control [35], which further supports the claim in references [30, 34] that social media influence by politicians has a negative impact. Reference [35] further raises concerns about data being misused by users on social media for political benefit and the need for added restrictions on social media to counter ill use of the platforms. Reference [44] supports the claim of reference [35] regarding data breaches and the need for better regulations regarding the usage of data.

Reference [32] states that the effect of social media on geopolitics is limited, and it simply serves as one tool among many as a force for political change. A similar point of view has been given by [45], while contradicting views are given in [46] where it is stated that social media can influence political outcomes significantly. Reference [32], however, mentions that geopolitics has an impact on social media rather than the other way around. Nonetheless, reference [32] also states social media has the capability to influence geopolitics but in a limited manner, as mentioned in reference [47].

According to Pauwels [37], although social has both positive and negative implications, the use of artificial intelligence to collect data from social media and manipulate the emotions and attitudes of other people is becoming more essential than hard power. Cybersecurity has become the priority of the world now and has significantly affected the geopolitics of the globe. Thus, we can say that the negative impact of social media on geopolitics is more prevalent. Moreover, the defence strategies in cyberspace need data-driven social media to improve the defence of nations. The negative impacts of social media manifest themselves in information overcontrol, information theft, and manipulation to sabotage other nations, information mercantilism, and the use of information as a strategic resource [38]. The impact of social media in creating unrest in society is contingent upon the hold of government on its institution and the powers to clamp down movements that influence geopolitics of the country [32].

Social media defends as well as challenges the existing world order. It influences traditional norms and values and replaces them with global networks and relationships. This is how social media negatively influences existing norms and threatens social setup. When global powers penetrate society through social media, the threat of local politics getting impotent increases. Moreover, geopolitical representations can alter indigenous politics through social media and serve the interests of other powers [33].

### 4.3. Social Media and Economic Growth

In the context of the link between social media and economic growth, according to [27], a participatory economy can induce economic growth due to the fact that more people get involved in contributing to the growth due to new opportunities created by social media. Reference [48] give a similar view as the one mentioned in [27], as the study discusses the prospect of participatory economic growth as a consequence of the increasing use of social media. The positive impact of social media can be highlighted by the fact that social media affect the larger economy and GDP of the country. Humans are always under social and psychological pressure to buy things that are unnecessary just because everyone else is buying those products. This group dynamics influence and shapes individual decisions in the presence of social media. Not only do mutual connections have impact on local decisions of buying, but also, due to the world as a global village, many trade agreements take place among countries due to social networking. Furthermore, [49] discusses the prospect of participatory labour through social media, which can induce better branding and economic growth for respective entities. Reference [49] also support the claims of [27] that the emergence of businesses from social media can be beneficial on the economic grounds, while it also has an impact on social relations and the well-being of individuals in a particular area.

As indicated earlier, social media has a significant positive impact on economic growth, contributing to the GDP of India and several European countries [28]. The reason behind the positive influence is that social media enables businesses to improve their product quality as well as product development planning. According to an estimate, 94% of all businesses use social media as their marketing tool. The use of social media causes economic growth due to cost reduction, effective feedback systems, and branding strategies. It leads to value addition in the products and an increase in revenue generation. According to [25], social media affects the economic growth of developed countries when governments intervene through more regulated social media campaigns for encouraging technology and so on. The role of government is central to economic growth due to social media. The authors of [28] also believe that the positive link between social media and economic growth is due to the fact that information exchange through social networks improves entrepreneurship and increases economic activities.

However, there are negative implications of social media as well. In the study of Dell'Anno et al. [18], it is identified that social media has a significant negative impact on economic growth; this finding is also portrayed in [36] and somewhat in [35] as it talks about negative economic growth for a particular sector. Reference [18] states that one of the reasons why the association between the two constructs is negative is because the productivity of the individuals can be affected poorly by social media. This claim is supported in reference [50], as the study mentions productivity as a challenge due to social media. It is observed that one of the prime reasons is the searching costs and the time invested by workers on networking reduces labour productivity [18].

Finally, in [36], it is found that social media and economic growth correlates; however, the relationship is negative as it has been observed that cities with fewer social media activity have better economic growth. The negative economic growth due to social media has also been discussed in the research by [18]. It has been discussed in the studies that a decrease in productivity due to social media causes negative economic growth.

## 5. Developing Artificial Intelligence and Cognitive Computing Tools to Mitigate the Risks

Social media is computer-mediated technologies with a huge amount of internet-based communication. Therefore, it generates a high risk for geopolitics and smooth economic growth from bad actors. AI and cognitive computing could help us mitigate those risks of social media. Following AI and cognitive computing tools can be used to address these issues.

### 5.1. Natural Language Processing (NLP)

NLP is the AI tool designed to process and analyze large amounts of natural language data. It can process information for speech recognition, sentiment analysis, and relationship extraction. Social media such as Facebook, Twitter, YouTube, and discussion forums uses this AI and ML tools to get demographic information, social interaction, emotions, and language use [28]. This tool can also be used to minimize the geopolitics risk. The Facebook team created DeepText software that allows analyzing the words of shared messages. The neural networking analyzes the sense of these words in order to evaluate the underlying meaning by relating with other words around it. DeepText software uses an AI algorithm to learn such words instead of a database for referencing [37]. It lets Facebook interpret words in around 20 different foreign languages by assigning every word to certain labels. On the other hand, Twitter introduces AI tools to recommend tweets from the timeline. This was achieved with the use of NLP, which enables the processing of thousands of tweets every second.

### 5.2. Facial Recognition System

It is another AI tool that can recognize or check a person from a digital picture or a video [38, 51]. For example, this tool can identify whether an individual was involved in a particular crime or just present at the scene. This tool has been used by several companies to investigate crime. Such as, Clearview AI has a vast database consisting of around 3 billion images that were collected from different websites such as Facebook, Twitter, Instagram, and YouTube. Clearview provides rights of more than 3 billion social media photos database to law enforcement agencies who can match any individual from those photographs. Trustwave is a leading global service provider that provides cybersecurity to companies for combating cybercrime, minimizing security risks, and securing data. Researchers of this company have developed an open-source platform named Social Mapper that enables facial recognition to monitor issues across social media networks. Researchers of different disciplines can use this open-source platform to detect issues that are creating risk for geopolitics and smooth economic growth by automatically locating social accounts based on a name and image on Facebook, Twitter, Instagram, LinkedIn, Snapchat, and other networks. Facebook also developed an AI tool named DeepFace that use two or more images to identify human faces. It also says that this algorithm identifies human faces more reliably than humans themselves with a 97% success rate. But their way of showing names on their faces has caused some concerns about the infringement of their freedom.

### 5.3. AI Tools to Identify Fake News

Fake and misleading data affect political, social, and economic relations. Especially, “fake news” gained global attention during the US presidential election in 2016, and researchers around the world are trying to develop new AI tools to identify fake news. According to [29], the top 20 fake news reports outperformed 3 months prior to the election through shares, responses, and reviews, and those fake news were from major news outlets. Facebook has often been blamed for promoting or encouraging vast amounts of “fake news” from a number of sources, including Russian agents seeking to manipulate US and European elections. To handle these fake news, Snopes created a web-based AI tool to help identify fake news; Hoaxy was designed to help users find fake news sites; and Le Decodex from Le Monde stores information in a database containing websites labeled as fake, real, and so on. CrowdTangle is a platform that helps monitor, discover, and analyze the social content early. Spike is a platform for finding and forecasting breakout and viral news. This platform analyzes thousands of news world data and forecasts what will drive interaction. Facebook has sophisticated algorithms that apparently recognize false or offensive news, inappropriate ads, or messages.

### 5.4. AI Tools for Detecting Hate Speech

Freedom of speech is the freedom to express ideas, opinions, thoughts, and ideas without restrictions. But this freedom gave way to hateful speech and social media can amplify conflict that creates a lot of geopolitical crises and harms economic growth. Thanks to the AI tolls that fired out those hateful speech anonymously [52]. In 2016, Google developed an AI algorithm that was designed to track and stop hate speech on the website and social media. Carnegie Mellon University researchers in Pennsylvania led by Dr. Ashique KhudaBukhsh have also created an AI algorithm that recognizes positive comments. This is an alternative approach to identifying and countering hate speech. Twitter utilizes the AI tool to recognize and eliminate accounts that have been used for hateful and racial tweets. So, in 2017, nearly 3 lacs terrorist-linked accounts were deleted using AI bots.

### 5.5. Fack ID on Social Media

Oxford Internet Institute recently has conducted a research and shown that misuse of social media is getting worse, especially by using fake IDs. Facebook used an AI algorithm recently removed thousands AI-generated profiles and accounts from the Facebook network [53]. Instagram used unethical practices to drive agendas for pro-Trump to around 55 million users. This platform utilized fake accounts with fake profile pictures created using AI to circulate polarizing, primarily right-wing information around the website, and even on YouTube and Twitter. Researchers around the world are trying to develop more sophisticated AI tools to identify fake IDs and fake profiles.

### 5.6. Cognitive Computing

Applying cognitive computing against massive data sets can help organizations process information more quickly and make smarter business decisions [54]. And cognitive computing is increasingly being used in the domain of risk management, mining often ambiguous and uncertain data to find indicators of known and unknown risks. Cognitive capabilities—including machine learning, natural language processing, and many other types of cognitive technology—provide a modern alternative to traditional analytics and are being applied to massive data sets to help find indicators of known and unknown risks.

## 6. Conclusions

Social media are online platforms that are able to facilitate the sharing and creation of career interests, ideas, and information, in addition to other forms of expression through networks and communities that are virtual, whereas geopolitics represents politics that is defined by geographical factors such as international relations. While economic growth can be defined as the increase in the financial means of a specific entity. Social media has seen a huge rise in users since the late 2000s decade, which has given rise to multiple opportunities and also risks. The discussion in the present study is based on the impact of social media on geopolitics and economic growth and the developing AI and cognitive computing tools to mitigate the risks.

It is identified through the studies that geopolitics is impacted by social media through the users' ability. Politicians can use social media to influence individuals by using certain strategies. Two strategies have linked populism theory to a politician's ability to influence individuals through social media. The ability to influence individuals through social media by politicians has been categorized as unethical and bad practice by multiple studies as the situation may lead to a conflict of interest at a later stage. Furthermore, it is identified that social media has given rise to the spread of news that is troublesome for geopolitics as some governments or organizations like to preserve the ability to censor content for their own benefit. Another implication identified by social media on geopolitics is the number of protests caused by the platforms. However, it is important to note that an opposite effect also occurs, that is, in the case of less censorship, there is a greater development of social media.

Regarding economic growth, it is stated in multiple studies that there is a significant and negative impact of social media on economic growth. The negative impact has been observed due to the fact that productivity level has decreased with the increasing usage of social media. Contradicting views, however, have been provided in other studies that have stated that there is a good opportunity through social media for having a participatory economy, which can be beneficial for countries. However, the mass development of social media coincided with the global financial crisis (2007–2009); thus, a spurious relationship between social media and economic growth may also exist.

It has been identified that social media has both positive and negative impacts on geopolitics and economic growth. Social media is able to unite diverse groups and individuals spread across the planet dedicated to specific issues. On the other hand, some argue that social sharing has encouraged people to use computers and mobile phones to express their concerns on social issues without actually having to engage actively with campaigns in real life. Their support is limited to pressing the “Like” button or sharing content. However, this thorough study ensures that the present study is valuable to academia and the relevant stakeholders to develop new theories and new AI and cognitive computing tools that can help mitigate the risks of social media for geopolitics to ensure smooth economic growth.

It is suggested for future researchers regarding the topic to analyze the impact of social media on censorship as there are still conflicting views on this subject and academia benefit from a well-constructed model on the impact of social media on censorship. Furthermore, it is suggested for future researchers conduct empirical research on social media's impact on economic growth with the use of relevant theories; it is found in the present study that the impact is negative, yet there is a conflicting points of view presented in other accessed material. Therefore, academia can find value in an empirical study related to the impact of social media on economic growth.

## Figures and Tables

**Figure 1:** PRISMA procedure.

**Table 1:** AMSTAR result.

AMSTAR 2 results	
The impact of social media on geopolitics and economic growth is a moderate quality review.	
(1) Did the research questions and inclusion criteria for the review include the components of PICO?	Yes
(2) Did the report of the review contain an explicit statement that the review methods were established prior to the conduct of the review and did the report justify any significant deviations from the protocol?	Yes
(3) Did the review authors explain their selection of the study designs for inclusion in the review?	Yes
(4) Did the review authors use a comprehensive literature search strategy?	Yes
(5) Did the review authors perform study selection in duplicate?	No
(6) Did the review authors perform data extraction in duplicate?	No
(7) Did the review authors provide a list of excluded studies and justify the exclusions?	Partial yes
(8) Did the review authors describe the included studies in adequate detail?	Yes
(9) Did the review authors use a satisfactory technique for assessing the risk of bias (RoB) in individual studies	Yes
(10) Did the review authors report on the sources of funding for the studies included in the review?	Yes
(11) Did the review authors account for RoB in individual studies when interpreting/discussing the results of the review?	Yes
(12) Did the review authors provide a satisfactory explanation for, and discussion of, any heterogeneity observed in the results of the review?	Yes
(13) Did the review authors report any potential sources of conflict of interest, including any funding they received for conducting the review?	Yes

**Table 2:** Systematic review.

Year	Title	Author (s)	Country	Findings
2013	Social media heightens political risks in emerging markets	Kay and Freely	USA	Governments must integrate social media into their strategies and recognize the political risk regarding social media. A comprehensive risk management plan regarding social media can prepare institutions with more ability regarding social media.
2013	The social media in the economy	Papachristou	Spain	The emergence of social media can produce economically benefitting results for some users. Furthermore, the study states that social media has laid foundations for a participatory economy, where one participant gains value from the action of others.
2016	Impact of social media on economic growth – evidence from social media	Dell'Anno et al.	Italy	After the tests, it is identified that social media has a significant and negative impact on economic growth. Further research suggestions included accessing whether the negative impact is due to greater consumption of nonmonetary content, decreased productivity, increased search costs, or a mix of the three factors.
2012	Social media - The new power of political influence	Auvinen	Belgium	Political opponents can use social media to learn from each other much more easily and openly.
2016	Infrastructures of empire: towards critical geopolitics of media and information studies	Aouragh and Chakravartty	United Kingdom	Social media has a strong impact on geopolitics as it exposes the current situation in locations where they might want to keep it a secret.
2016	The geopolitics of social media in Eurasia	Chausovsky	Russia	The use of social media has been shaped by geopolitical circumstances, rather than the other way around. Certainly, social media can act—and has acted—as an enabler of significant political developments. But, far from causing revolutions—and more importantly—ushering in regime change following these revolutions, social media simply serves as one tool among many as a force for political change.
2019	Digital communication disrupting hegemonic power in global geopolitics	Simons	Sweden	Social media and new media are playing a greater part in international relations and politics. They are being used as a means to defend the existing world order and as a means to undermine it. These new forms of media are potentially very potent instruments of influencing the course and discussions on the existing world order and its possible directions. They are able to unite diverse groups and individuals spread across the planet dedicated to specific issues.
2016	Populism and social media: How politicians spread a fragmented ideology	Engesser et al.	Switzerland	The paper states that social media gives populist politicians and other key figures the ability to voice out their opinions and gain a following, while the study explores deep into populism culture and suggests refined structuring of the topic for the future.
2019	What to do about social media? Politics, populism and journalism	Crilley and Gillespie	United Kingdom	Lack of accountability from social media outlets can cause the political use of social media to be out of control. The political use of social media platforms is conducted on unethical grounds and should be subject to appropriate restrictions.
2019	E-capital and economic growth in European metropolitan areas	Kiuru and Inkinen	Finland	There is a relationship between economic growth and social media; however, the relationship is negative as it has been observed that cities with fewer social media activities have better growth economically.
2016	The role of social media and its implication on economic growth on society in India	Sharma	India	The use of social media causes economic growth due to cost reduction, effective feedback systems, and branding strategies.
2016	Development impact of social media	Ackland and Tanaka	Australia	Social media impacts the economic growth of developed countries when governments intervene through more regulated social media campaigns.
2018	The influence of entrepreneurship and social networks on economic growth	Chen et al.	China	There is a significant positive influence of social networks on economic growth.
2019	The new geopolitics of converging risks	Pauwels	USA	Social media is reshaping the geopolitics in both positive as well as negative dimensions.
2019	The geopolitics of information	Rosenbach and Mansted	USA	In terms of geopolitics, social media has both pros and cons in modern societies; however, the negative consequences are prevalent.

## Data Availability

The data supporting the findings of this work are available within the article.
